The article "Ethnobotanical and conservation studies of tree flora of Shiwalik mountainous range of District Bhimber Azad Jammu and Kashmir, Pakistan" was retracted in 2023. Reasons: a conflict of interest; concerns about the peer review; concerns about the authorship.

# Ethnobotanical and conservation studies of tree flora of Shiwalik mountainous range of District Bhimber Azad Jammu and Kashmir, Pakistan

**DOI:** 10.1371/journal.pone.0262338

**Published:** 2022-02-07

**Authors:** Humaira Khanum, Muhammad Ishtiaq, Khizar Hayat Bhatti, Iqbal Hussain, Muhammad Azeem, Mehwish Maqbool, Tanveer Hussain, Waheeda Mushtaq, Sumaira Thind, Rohina Bashir, Mahnoor Muzamil, Shams H. Abdel-Hafez, Samy Sayed

**Affiliations:** 1 Department of Botany, Mirpur University of Science & Technology (MUST), Mirpur (AJK), Pakistan; 2 Department of Botany, University of Gujrat, Gujrat City, Pakistan; 3 Department of Botany, Government College University Faisalabad, Faisalabad, Pakistan; 4 Department of Chemistry, College of Science, Taif University, Taif, Saudi Arabia; 5 Department of Science and Technology, University College-Ranyah, Taif University, Taif, Saudi Arabia; King Khalid University, SAUDI ARABIA

## Abstract

The present study was carried out to explore and document traditional ethnobotanical knowledge of indigenous rural communities of Shiwalik mountainous range regarding tree flora of the area, District Bhimber of Azad Jammu and Kashmir, Pakistan. The local people of the area primarily depend on wild flora for life sustenance and cure of different infirmities. In this research, data was collected through visual appraisal and participatory rural approach using questionnaire method by applying semi-structured and structured-interview protocols (S4 Table). To validate and explore novelty of research work, various quantitative ethnobotanical indices like informant consensus factor, use value index, fidelity level, relative frequency of citation, relative importance of plants, rank order of priority, Jaccard index and priority ranking were used. The highest ICF was found for jaundice with 0.91 value followed by ICF values of 0.89, 0.86 and 0.85 for wounds, skin diseases and stomach pains, respectively. Fidelity level predicted that *Azadirachta indica* (Indian lilac tree) ranked first (100%) for its prevalent use in ethnomedicines. Highest use value index (0.61) was found for *Azadirachta indica* while the highest relative frequency of citation (55) was measured for *Melia azedarach*. The relative order of priority index was the highest for *Azadirachta indica* and *Acacia arabica* L. (ROP = 100) depicting their prevalent use in ethnomedicines. For EB study, the highest relative importance (50.8) was found for *Azadirachta indica* with good number of agro-uses and its seeds and bark are sold or marketed in local markets to prepare herbal therapeutics by indigenous practioners. The Jaccard index depicted that many traditional ethnomedicinal uses of prescribed trees were novel in recipe form or first time reported such as *Senegalia modesta* (Phulai) resin was used to prepare ‘Panjoori’ a local tonic prepared from cow or buffalo butter mixing with seeds *of Papaver somnifera* (Kashkhash) and *Prunus amygdalus* (Badaam). The wood of many trees like *Pinus roxburghii* (pine), *Dalbergia sissoo* (rosewood), *Senegalia modesta* (Phulai), *Acacia*. *Arabica* (kikar), *Bombax cieba* (cotton tree) is commercially sold as timber in markets (S3 Table). The research proved that population explosion and climate changes have triggered severe biotic and abiotic pressure on tree flora of the study area of Bhimber, AJK. The research describes that plants like *Terminalia belerica* (belerica), *Terminalia arjuna* (arjun tree), *Cassia fistula* (Indian laburnum), *Butea monosperma* (bastard teak), *Phyllanthus emblica* (Indian gooseberry), *Morus laevigata* (Shah toot), *Bauhinia variegata* (orchid tree) and *Flacourtia indica* (Indian plum/ kakoo) are threatened species and their population is highly reduced and if reclamation measures for their conservation are not taken, it may lead towards their complete loss from the area. This research recommends sustainable ethnobotanical use of tree flora, their growth and conservation for green and ecofriendly environment for safe and secure future of human generation.

## Introduction

Plants being autotrophic acts as primary source of nutrition on earth. All other life forms depend directly or indirectly on plants for various purposes [1]. Since emergence of life on earth plants are being used for various purposes: food provision, fodder/feed for animals, an aesthetic environment, medicinal source, shelter and other byproducts such as fibers, drugs, oils, latex, pigments and resins for sustenance of life [2]. Plants maintain the balance of nature for continuation of life on earth and study of plants is named as “Ethnobotany” coined by John Hershberger in 1896, pertaining to study of “the plants used by the primitive and aboriginal people” [3, 4].

Botanical or herbal medicines are extensively used in different traditional health care systems to cure numerous diseases [5–7]. About 50,000 angiosperm plants are being used world widely as medicinal plants as reported by Schippmann *et al*., [8]. It is narrated that herbal medicines are used in powder, extract, decoction, infusion, tea, tincture, paste, balm and poultice form [9]. According to an estimate about 80% of world’s population residing in developing countries prevalently use traditional herbal medicines to cure different infirmities [10]. The non-medicinal uses of plants like: fuelwood, fodder, forage, hedging, furniture, construction, weapon, home utensils and aesthetics are of also paramount in life of human being. Such uses of medicines and other forms are referred as ‘Ethnobotany’. The relationship of plants diversity and cultural diversity has significant correlationship and plants play pivotal role in life of man [11].

Among plants, trees have great significance in ecosystem and provide multifarious uses for local people of any area in world such as fuelwood, shadow, agriculture tools, furniture, house-making, decoration, war-tools, fodder, forage, medicines and fruits as food etc [12, 13]. Trees are key pillars of any ecosystem as being main producers as well as indicators and protector for the other plant species i.e. shrub and herbs as under storey in forest which is inevitable for faunal biodiversity [14, 15]. Trees provide many other non-timber forest products (NTFPs) uses and hence also significant part of habitat or ecosphere characterization depends on tree population and diversity. The uses of trees for drug discovery and development is also of high worth in pharmacological industries [16]. Without tree diversity, life biodiversity on land seems rare or scare and even very difficult or impossible, so study of trees uses and their population structure and conservation is very inevitable [17, 18].

Trees are primarily used in different herbal drugs in different areas of country [19]. The extensive use of root, flower, seeds, bark and leaf of trees has created threat for many tree species which lead towards threatened or rare paradigm which demands urgent need of conservation many tree species. The territory of Azad Jammu and Kashmir is located in eastern and northern side of Pakistan which is connected with Punjab and KPK provinces. Area of Azad Kashmir due to its phytogeographic location and religious paradigm is prime worth; the indigenous communities of AJK have strong cultural and ancestral family links with various ethnic communities of adjoining areas of Pakistan which makes this area also very interesting because of its diverse bioculture (Fig 1). History depicts that routes of Kashmiris are linked to ancient Indo-Ayran ethnic group “Dardic” habitants of eastern Afghan border and northern parts of Pakistan and India. As District Bhimber serves as a gateway between Azad Kashmir and Punjab due to which it is popularly known as ‘Bab-e-Kashmir’ meaning “door to Kashmir” [1, 18]. The common traditional ethnic groups of the study area are: Jat, Mirza, Malik, Rajpoot, Bhatti, Sheikh, Syed, Awan and Gujar. The prevalently spoken languages are Urdu, English, Dogri, Kashmiri, Potohari and Saraiki which are variable [1, 18]. The common professions of indigenous inhabitants of SMR area are: farmer, woodcutter, carpenter, forest protector, herbalist (hakeem), nomadic tribes, honey bee keeper, mason, labour men, while some are servants in Govt and private sector (Fig 2). Majority of local people of the area primarily depends on natural resources as for livelihood earnings from trees or their byproducts. The specific geographic location of area, rich cultural and biological diversity makes the area unique and interesting hence, it is selected for ethnobotanical research. The previous ethnobotanical research works conducted on District Bhimber and other areas of AJK have revealed wild flora particularly trees are the mostly affected due to fuelwood collection, over grazing, fire, expansion of silviculture, over harvesting of trees’ leaf for forage, timber mafia act of ruthless cutting has been cause of phytodiversity loss in many areas of world [20–26] and in the study area tree flora is ruthlessly harvested which may culminate in same fate.

**Fig 1:** Map of study of Shiwalik mountaineous range of District Bhimber of Azad Jammu and Kashmir, Pakistan.

**Fig 2:** Demographic information of Study area Shiwalik mountaineous range of District Bhimber of AJK.

### Rationale of study

The study area comprises of mountaineous terrains with rich cultural and phytodiversity which is unique and hitherto it is not explored. Tree flora is very prominent in the study area in *Pinus* forest and *Acacia* scrub forest which provide many provisional and regulatory ecosystem services to indigenous people of the area. Tree layer is dominant layer which controls other layers of the forest. Due to exponential increase in population of human being, people use these trees for multipurpose to meet necessities of daily which is creating drastic biotic pressure on tree flora of the area.

So the ethnobotanical data compilation on tree species will be important for future research and conservation work to be carried by indigenous people and forest Department. This makes rationale of the ethnobotanical study in the study is of paramount significance. Albeit many ethnobotanical studies are conducted in AJK [27–30], others areas of country [31–33] and District Bhimber of AJK [34–36], but hitherto no quantitative ethnobotanical research is conducted on tree flora of Shiwalik mountain range of District Bhimber. This study is novel work which provides baseline studies on tree flora of the Bhimber mountaineous zone which will be useful in novel drug discovery and formation of many essential products of life which demands their conservation for sustainable use and availability for future generations.

### Research objectives

The current research study is conducted on tree flora of Shiwalik mountaineous range of District Bhimber (AJK) with multifarious objectives: (i) to collect and document traditional ethnobotanical knowledge of tree flora, (ii) to validate authenticity of collected data using quantitative statistical tools to explore highly potential medicinal trees for novel drug discovery through dedicated ethnopharmacological approaches and (iii) to determine causes of pressure on tree flora and their conservation status with provident recommendations to mitigate and eradicate it cause of tree diversity.

## Materials and methodologies

### Description of study area

Phytogeographically state of Azad Jammu Kashmir state is located in northern region of Pakistan occurring in lap of northern Himalaya mountain range. The territory of AJK as an area of 13,297 km^2^ with high lofty mountains, incessant hilly terrains and torrents (Fig 1). The study area (Shiwalik mountain range) of District Bhimber lies within 33°50′36″N and 73°51′05″E [37]. These mountains are extension of Shiwalik mountainous range starting from northeast of Nepal and India, entering in Pakistan from northern side. The soil of study area is mostly acidic and sandy-clay with supporting specific type of rich floral and faunal biodiversity [38].

### Ethnobotanical data compilation and authentication

Ethnobotanical data of tree flora was collected from local people inhabitating in different villages of Shiwalik mountaineous range, fuelwood and timber sale points from District Bhimber during 2015–17. Data was collected through several field visits using visual appraisal assessment and rapid rural appraisal (RAA) method employing questionnaire proforma. The field trips were organized in different seasons to cover maximum cultural and tree phytodiversity of all sampling sites (villages and markets sale points) of the area. In visual appraisal assessment (VAA) method, data was collected through personal observations made during field visits from wild areas, markets, farms, fields, wooden handicraft shops and community houses by seeking permission from village representative and/ or from house owner. In RRA method, data was collected from 190 respondents using questionnaire proforma employing open-ended interview and close-ended interviews procedure following protocol of Ishtiaq *et al*., [1, 18]. The respondents were old-age inhabitants, farmers, fuelwood cutter, timber wood stockists, carpenters, industrialists, women, mid-wives, herbalists (hakeems), nomadic tribes (bakarwals) and herd-owners (shepherds).

In the interview process, plants were categorized according to use-form such as “food, fodder, thatching, hedging, shelter, fuelwood, timber”, their subsequent economic value and other relevant purposes were recorded. In field trips, plants were collected (having flowers, fruit or both) pressed, dried, preserved and mounted on herbarium sheets by incorporating voucher numbers (MUH-) which were deposited in herbarium of Department of Botany Mirpur University of Science and Technology (MUST) Mirpur-10250 (AJK) Pakistan for future reference. The collected plants were identified by taxonomist (Dr. Muhammad Ishtiaq) and were crossed checked with Flora of Pakistan (booklets), online flora of Pakistan (www.efloras.org) and plant list website (www.theplantlist.org) for proper authentication of botanical names and families [39].

### Ethical statement

The permission for field study and collection of wild plants (trees) from wild and Forest areas of Shiwalik Mountian Range (SMR) zones of District Bhimber (AJK) was obtained from Departmental ethical committee (DEC) on official letter (Ref No: 31/DEC/BOT/2015; Date: 20/06/2015) and counter signed by Head of Department.

### Field survey permission letter

An official field permit (Ref No: DFO/655/2015 Dated: 01/07/2015) was obtained from District Forest Officer (DFO) to make field visits of forest area of SMR of Bhimber and to collect samples from plants (trees). The right of obedience of forest rules was fully followed as per SOPs provided by the relevant office and guidance of DEC was also fully obeyed.

### Quantitative analysis

The collected data was organized in tabular form for further statistical analysis. For validation and authentication of collected ethnobotanical and ethnomedicinal data, different standard quantitative ethnobotanical indices were employed [40–45]. For analysis, informant consensus factor, fidelity level, relative importance of plant, use value index, relative frequency of citation, relative popularity level and rank order of priority were used according to procedures of previous researchers [1, 9, 46, 47].

#### Informant consensus factor (ICF)

ICF analysis was carried out for each category or group of diseases to determine the consensus of informants on the reported ‘ethnomedicinal uses’ for the group of diseases and later on various infirmities were categorized in different categories [1, 12]. ICF was calculated using following formula:

$$ICF=\frac{Nur-Nt}{Nur-1}$$

where, ‘Nur’ represents number of use citations minus (-), ‘Nt’ total number of plant species used cited by respondents; divided (/) by the number of use citations in each category minus one [9, 46, 47]. If the result is nearer to (1) or exactly (1) then reported plant species is abundantly used by locals. Whereas, if value is near to (0) or comes out to be zero then reported plant species is casually used or not used by inhabitants of area [1, 12].

#### Fidelity level (FL)

The fidelity level of the data was calculated which depicts the percentage (%age) of interviewees claiming any use of a particular plant for the same major purpose or field and total number of commonly reported usages or ailments. It was calculated according to formula:

$$FL\;(\%)=\frac{Np}{N}x\;100$$

where; ‘Np’ depicts number of informants who claimed a particular use of a plant species used for a typical disease and ‘N’ means that number of informants/interviewees who used the plants as an ethnomedicine to treat given diseases [1, 12].

#### Relative popularity level (RPL)

RPL describes the frequency use of a particular species. In some analysis sporadically FL provides same usage frequency of various species then Relative popularity level index is used to reassure and confirm FL values of various trial species. RPL value generally ranges in-between 0–1, where value 1 or nearer value to 1 represents maximum RPL value while 0 or nearer to 0 represents minimum value frequency for particular disease [12, 39]. Value of RPL increases in accordance with informants as it rises correlation coefficient factor r = 0.10. For example, if a particular species is reported by 25 or more individuals it will have high RPL value and vice versa. RPL is calculated by proportion of (I_u_ /number of individuals reported the use of particular plant). When 25 of more individuals report for a particular species RPL value becomes (I_u_/12) which gives one (1) and specie is ranked as Popular (P). Whereas if less than 25 individuals report plants uses then respected plant species is ranked as unpopular (UP) [12, 39]. Marginal value in-between, P and UP of particular plant refers point where further increase in number of informants don’t upswing medicinal use per plant species.

#### Rank order popularity (ROP)

To determine correction between FL and RPL, rank order popularity is used. ROP designate the popularity rank to individual in accordance to FL and RPL values. Following formula is used for ROP

ROP=FLxRPL (i)

ROP value represents higest rank/level for popularity of various MPs used to cure specific disorder [12, 39] RPL and ROP statistical test are significantly important for determining EB importance of commonly used plant in respected area.

#### Relative importance of plant (RIP)

To determine the pharmacological or pharmaceutical significance of individual plant relative importance of plants (RIP) was used following protocol of Umair and Amjad [1, 25].

$$\mathrm{RIP}=\frac{\mathrm{Rel}.\;\mathrm{Ph}+\mathrm{Rel}.\;B.S.}{2}\times 100$$

whereas Ph. is pharmacological features of the plants and Rel. Ph: relative pharmacological importance; rel. BS: body system treated. The relative Pharmacological significance can be caluclated by the given below formula [12, 25].

$$\mathrm{rel}.\mathrm{Ph}.=\frac{\mathrm{Ph}.\;\mathrm{of}\;\mathrm{given}\;\mathrm{Plant}}{\mathrm{Ph}\;\mathrm{of}\;\mathrm{all}\;\mathrm{reported}\;\mathrm{plant}\;\mathrm{species}}$$

whereas Ph. is pharmacological attributes of the each provided plant and rel. Ph. is the relative number of pharmacological properties referenced for an individual plant.


$$\mathrm{rel}.\mathrm{BS}.=\frac{\mathrm{BS}\;\mathrm{of}\;\mathrm{given}\;\mathrm{Plant}}{\mathrm{BS}\;\mathrm{of}\;\mathrm{all}\;\mathrm{reported}\;\mathrm{plant}\;\mathrm{species}}$$

Here BS is the number of body System healed by single plant species whereas, rel. BS is total relative number of body system treated by the given plant species [1, 12].

#### Use value index (UVI)

The use value index (UVI) demarcates relative importance of different uses of the specific species. It was determined by using past cited formula following protocol of previous researchers [12, 25].


$$UV_{i}=\frac{\sum Ui}{N}$$

Whereas UV indicates “relative use value” of the single species; “U” is the ‘number of uses mentioned by each informant for the species and “N” is the ‘total number of informants who reported that species [25].

#### Relative frequency of citation (RFC)

Relative frequency of citation is used an index to explore significance or importance of each species occurring in the local area. RFC was determined by “dividing the number of informants” confirming the frequency of citation (FC) by “total number of informants” who participated in survey according formula of [12, 26, 39].


$$RCF=\frac{FC}{N}R$$

Where, ‘0 < RFC >1’; and FC is the ‘number of informants’ reporting use of a particular species and N is the ‘total number of informants’ involved in study survey.

#### Priority ranking (PR)

Priority ranking (PR) method was used for indicating the preference of the local people about the potential use of each plant in certain use and it describes the biotic pressure on the plants of the area and it assist to calculate the conservation status of various species in the study area [12, 25].

#### Jaccard Index (JI)

The JI was used to find out novelty of ethnobotanical study which was conducted on tree flora of SMR of District Bhimber of AJK. This index compares EB data of current study with previously conducted ethnobotanical expeditions in other parts of AJK, Pakistan and world and similar the rationale used for “indigenous communities in study areas”. The JI was calculated using formula of González-Tejero *et al*., [12] JI = c×100/a+b-c; where ‘a’ means number of tree species found in study are ‘A’; while ‘b’ is details of tree species found in area ‘B’ and c is number of species commonly present in both areas or reported by both communities ‘A’ and ‘B’.

## Results and discussion

### Rationale of research study

The plants are very important part of biosphere and have essential role in life of man. All people of world are dependent on plants for oxygen, food, fibers, drugs, oils, latex, pigments and resins which is inevitable for sustenance of life [12, 25]. The current research was conducted to study role of tree species of Shiwalik mountain range (SMR) of District Bhimber of AJK, Pakistan in forest ecosystem and life of indigenous people of the area. The hypothesis was based on that theme that “*whether without trees ecosystem of forest and life of mankind of SMR can have survival*?” and *“is ethnobotanical study useful for analysis of conservation of tree flora of the study area*? As trees are key producers and dominating part of any terrestrial forest ecosystem, hence their ethnobotanical study and conservation analysis is conducted and presented with prospective recommendation.

### Demographic characteristics of respondents

The study comprises of domestic or commercial uses of tree flora of SMR of District Bhimber of AJK in which 35 plants have been reported by 190 informants (105 males, 85 female). Informants including three broad categories (i) 90 indigenous community people (ICP), (ii) 70 traditional herbal practioners (THPs) and (iii) 30 wood selling people (WSP) from randomly selected different villages and local markets. The demographic information is presented in different fractions as shown in Fig 2. In the survey it was explored that male community is directly linked with tree flora as they cut, transport and sale tree in form of fuelwood, fruits and timber in local and national markets [12, 26]. In ethnomedicinal survey, it was found that mostly elder people have more information of TEMs than youth as it may be due to corrosion of TEMs in young generation with advent of technology and easy availability of allopathic drugs [12, 30]. Furthermore, it was concluded from results data that female communities have more traditional ethnobotanical information about wild flora [12, 26] than male but not significant difference as cited in past works [3, 18, 30, 31] and this might be due reason that both male and female work in forest and home as farmer, shepherd and cattle herd-man.

The local people use wild medicinal plants (WMPs) not only at their own homes as food phytonyms and tonics but also sale to herbal doctors (hakeem) and local markets traders to earn money. It was also found that old people have more information about the MPs and TEMs than young community because they spent long time with their ancestors (Fig 2) and used TEMs for disease cure [12, 45]. It was noted that hakeem (traditional herbalists) having 10–15 years experience possessed the highest (33%) level of traditional ethnomedicinal knowledge. It was found that illiterate people of study area have more information of TEMs because they follow traditional cultural rituals more prevalently with great passion and belief than educated inhabitants [12, 26]. A common trend of decline in TEK and TEMs use was seen in high literate people that may be due to fact that literate people prefer to use allopathic medicines because they can afford to buy these medicines and prefer prompt relief from infirmities. In contrast to this, indigenous old and illiterate communities prevalently have more TEK and use of TEMs because they believe that WMPs have no toxic effects and possess strong curing power. The botanic drugs are hitherto used in various areas of world [16, 17, 21] Pakistan [9, 20, 28, 44] and particularly in Azad Jammu and Kashmir due to mountaineous and rural geographic bonded with traditional cultures [1, 3, 6, 12, 15]. It is generally cited in different researches that female community possess more knowledge than men because they are in touch with plants in daily life but female are mostly shy, religiously restricted and less participant in of interview due to cultural ban. To cope this issues an indigenous female translator was hired to communicate with rural women of area for gathering maximum TEMs knowledge following perception of Amjad *et al*., [27, 40].

### Distribution pattern, collection, identification and preservation

In the investigated area, information of 35 tree species belonging to 17 families were recorded, gathered from different sampling sites: villages, timber stocks, sale points and furniture industries of District Bhimber of AJK. It was explored that north facing mountains rich population diversity than south facing which might be due to high altitude, moisture content and humidity is generally higher in north facing hills. The collected plants’ sample were bearing flower or fruit or both which were used for identified using standard protocols as described in above methodology section. The dried and prepared specimens were submitted in Herbarium (with code of MUH-), Department of Botany bearing valid voucher numbers for future reference and study [31, 45]. The floristic profile of wild indigenous plants (WIPs) was prepared comprising of family name, habit (herb, shrub or tree) and local name of each plant (S1 Table).

The distribution pattern depicted that trees of Moraceae and Mimosaceae were dominant with 07 and 06 species, respectively. Meliaceae, Rhamnaceae and Meliaceae with 04, 03 and 02 species, respectively. Most of the trees were used as fuelwood along with other uses such as food (fruit/vegetable), fodder, house construction, honey bee plants, making sports goods, fencing, in making of agricultural tools, and thatching for cattle herd sheds or mud houses. Ethnobotanical data collected from study area depicted that *Dalbergia sissoo* Roxb., *Bauhinia variegata* L. and *Azadirachta indica* A. Juss. possess multiple uses such for fuelwood, timber, fodder and shelter forming. The multiple use of trees by the local people causes severe biotic pressure on it this has lead towards to threatening of many species. It was concluded that *Butea monosperma*, *Terminalia belerica*, *Terminalia chebula*, *Cassia fistula* and *Cedrela toona* was under high conservation threats and these outcomes were found in-line with previous works [12, 18, 20]. They recorded respected trees with high usage percentage by local inhabitant for various purposes such as fuel, fodder, furniture, timber, medicinal and vegetable in Shakagarh, District Narowal, Pakistan.

It was found that 18 tree species were used in different TEMs to cure fever in various local ethnic communities. While four tree taxa are reported to be used in sex cure or sex booster prevailing in different TEMs of study area. 16 trees’ parts are declared to be used in cure of wound healing and wound pain analgesic agent. Similar research has been reported in previous studies that trees are commonly used for cure or relief of wound or wound pain [12, 20, 26]. In this study, it was found that one tree (*Ziziphus* genus) was used for curing of snake sting pain and poison. The plant *Butea monosperma* and *Ficus auriculata* is used as wormicide to treat of stomachache and intestinal infections. It was found the commonly prevailing diseases diabetes is predominantly treated by using green medicines obtained from *Eugenia jambolana*, *Ficus bengalensis*, *F*. *palmata* and *Emblica officinalis*. The data analysis depicted that Moraceae ranked 1^st^ with 22%, Mimosaceae was 2^nd^ number with 17% and Meliaceae ranked at 3^rd^ with 11% of share in total studied taxa of trees (Table 1). These results showed that Morus and other trees of this family are more prevalent in the area than other trees of families. These results are congruent with previous work of Mehwish *et al*., [13, 30].

**Table 1:** Family index of trees of Shiwalik Mountain Range of District Bhimber Azad Jammu and Kashmir, Pakistan.

Sr No.	Families	No. of Species	%age of Species
01	Anacardiaceae	01	3%
02	Arecaceae	01	3%
03	Bignoniaceae	01	3%
04	Bombacaceae	01	3%
05	Euphorbiaceae	01	3%
06	Meliaceae	04	11%
07	Mimosaceae	06	17%
08	Moraceae	08	22%
09	Myrtaceae	02	5%
10	Malvaceae	01	3%
11	Papilionaceae	02	5%
12	Polygonaceae	01	3%
13	Pinaceae	01	3%
14	Rhamnaceae	03	8%
15	Simaroubaceae	01	3%
16	Tiliaceae	01	3%

### Various ethnobotanical use forms of tree flora

Plants have been extensively used for various purposes by man since their existences. Some of common purposes for which plants are being extensively used in study area are listed in Table 2. About (19%) plants are used as fodder, (31%) for timber, (17%) for fuel, (8%) for making goods, (12%) for construction purposes, (2%) for bee boxing, (9%) as insect repellents and (9%) for veterinary medicines (Fig 3, S1 Table).

**Fig 3:** Percentage contribution of different plants for EB/ EM purposes from SMR of District Bhimber AJK, Pakistan.

**Table 2:** ICF value of ethnobotanical uses of tree plants of SRM of District Bhimber AJK, Pakistan.

Sr. No	Categories	No. of species(nt)	%age of species	No. of Use citation (nur)	$ICF=\frac{nur-nt}{nur-1}$
01	Timber	10	16.39	20	0.53
02	Fuelwood	11	18.03	15	0.29
03	Goods	09	14.75	17	0.50
04	Construction	10	16.39	11	0.10
05	Fodder	09	14.75	21	0.60
06	Bee Boxing	05	8.20	9	0.50
07	Agricultural tools	04	6.56	12	0.73
08	Wheat threshing	03	4.93	8	0.71
	Total	61	100	113	3.96

### Informant consensus factor of ethnobotanical uses of trees

The informant consensus factor (ICF) was calculated to evaluate different ethnobotanical uses of different plant species reported during course of field research. For calculation of ICF; various EB uses were classified into 6 groups: fodder, fuel, construction, furniture, making goods and decoration as per uses reported by locals (Table 2; S1 Table). ICF results showed that mostly plant sources are used for timber and fodder with first rank, followed by wood used for fuel and construction purposes moreover, for various goods and veterinary purposes (Table 2). While lower ICF values were calculated for uses like basket making, wheat threshing, agricultural tools, roti maker and wild edible fruit.

### Informant consensus factor of diseases occurrence and ethnomedicinal uses

The major aliments were classified into 13 disease categories by using ICF index parameter. According to ICF values the highest numbers of plant species were used against skin diseases, eye diseases and asthma (Table 3; S1 Table) which indicates common prevalence of these infirmities in the study area. That may be due to common exposure of indigenous in wild areas and fields as they have to do work for their house tasks. The ICF analysis depicted that mostly prevailing diseases in SMR area were fever, cough, wounds, jaundice, stomachache, diarrhea and kidney disorders. The highest ICF was found jaundice with 0.91 value followed by ICF values of 0.89, 0.86 and 0.85 for wounds, skin diseases and stomach pains, respectively. This high ratio of prevalence of these infirmities may be due to fact that study area is remote and hilly where indigenous people mostly lack basic facilities of life and there is scarcity of western medicines drugs. Wounds occurrence ratio in SMR area was found very high because local people are always working in forest and hilly torrents to conduct their farmer relevant activities. Due to high intensity of facing outside or open air in dust or cutting of grasses causes skin allergy or skin infirmities. These findings are congruent with previous works of conducted in different areas of country on ethnobotanical studies [1, 13, 31]. The least value (0.55) of ICF was found for diabetes which is due to highly active life of indigenous people in which food is burnt and no excessive calories are retained, hence no diabetes is seen in rural or hilly workers or inhabitants in different areas of world [1, 25, 31].

**Table 3:** ICF value of ethnomedicinal uses of trees of Shiwalik mountaineous range of District Bhimber AJK, Pakistan.

S No	Categories	No. of species(nt)	%age of species	No. of Use citation (nur)	$ICF=\frac{nur-nt}{nur-1}$
01	Skin diseases	04	5.33	22	0.86
02	Wound healing	08	10.67	67	0.89
03	Fever	09	12.00	73	0.89
04	Stomach diseases	09	12.00	55	0.85
05	Cough curing	06	8.00	33	0.84
06	Cancer	04	5.33	11	0.70
07	Jaundice	06	8.00	54	0.91
08	Asthma	03	4.00	13	0.83
09	Diarrhea	07	9.33	22	0.71
10	Diabetes	06	8.00	12	0.55
11	Kidney diseases	04	5.33	15	0.79
12	Eye diseases	03	4.00	9	0.75
13	Tooth problems	06	8.00	7	0.17

### Relative frequency citation (RFC) and use value (UV) of ethnobotanical uses trees

Ethnobotanical significance of various plants was calculated by using relative frequency of citation (RFC) and use value (UV). RFC and UVI indices were used to find out the medicinal potential of different tree taxa and future prospective for pharmacological research and novel drug discovery with subsequent drug development. RFC analysis confirms that indicated plants *Melia azedarach*, *M*. *Azadirachta*, *Senegalia modesta* and *Butea monosperma* have good role as TEMs in curing of various chronic or acute infirmities in study area (S1 Table). RFC confirmed the medicinal importance and acceptability of MPs with frequency of citations in the study area to cure various diseases. The RFC of medicinal plants species of the study area ranged from 18 to 55 (Table 3). RFC and UVi was calculated for ethnomedicinal and ethnobotanical potential uses and whose values in tabular is presented in matrix form (Tables 4, 5).

**Table 4:** Relative frequency of citation (RFC) and use value (UV) and of different important EB plants from SMR District Bhimber AJK, Pakistan.

Sr. No.	Names of plants	Common name	Family	Ethnobotanical Use	RF	RFC	UV	UVi
						65 informants participated in analysis		
01.	*Acacia arabica* L.	Kikar	Mimosaceae	Wood	43	0.66	23	0.35
02.	*Acacia nilotica* (Linn.) Delile.	Jangle Kikar	Mimosaceae	Wood	39	0.60	42	0.65
03.	*Ailanthus altissima* (Mill.) Swingle	Toon	Simaroubaceae	Wood	38	0.58	33	0.51
04.	*Albizia julibrissin* Durazz.	Jangle shree	Mimosaceae	Wood and for goods	27	0.42	16	0.25
05.	*Albizia lebbeck* L.	Shree	Mimosaceae	Fodder, wood	33	0.51	21	0.32
06.	*Albizia procera* L.	White shree	Mimosaceae	Basket making, wood, fodder.	29	0.45	25	0.38
07.	*Azadirachta indica* (A.) Juss.	Neem	Meliaceae	Wood, fodder	55	0.85	35	0.54
08.	*Bombax ceiba* L	Simbal	Bombacaceae	Cotton and wood.	40	0.62	55	0.85
09.	*Broussonetia papyrifera* L.	jangle toot	Moraceae	Wood, fodder	52	0.80	31	0.48
10.	*Butea monosperma*	Chechra	Papilionaceae	Wood, fodder	42	0.65	54	0.83
11.	*Cedrela toona* Roxb.	Cedar	Meliaceae	Wood, fodder	38	0.58	33	0.51
12.	*Dalbergia sissoo* L.	Tali	Papilionaceae	Timber	25	0.38	59	0.91
13.	*Emblica officinalis* L.	Amala	Euphorbiaceae	Making soap and shampoo, wood	31	0.48	45	0.69
14.	*Eucalyptus citriodora*	Safada	Myrtaceae	Wood	39	0.60	43	0.66
15.	*Eugenia jambolana* L.	Jaman	Myrtaceae	Fruit, wood	19	0.29	28	0.43
16.	*Ficus bengalensis* L.	Bohrr	Moraceae	Fruit, fodder, Wood	34	0.52	45	0.69
17.	*Ficus elastica* Roxb.	Rubber	Moraceae	Fruit, fodder, Wood	20	0.31	43	0.66
18.	*Ficus palmata* Forssk.	Phagwar	Moraceae	Fruit, fodder, Wood	22	0.34	32	0.49
19.	*Ficus religiosa* L.	Pipal	Moraceae	Fuirt, fodder, Wood, thatching	24	0.37	31	0.48
20	*Melia azedarach* (L.) Pers.	Darik	Meliaceae	Seed, fodder, Wood, fodder	24	0.37	46	0.71
21	*Ziziphus mauritiana* Lam	Jandi	Rhamnaceae	Wood, fruit, fodder	18	0.28	38	0.58

**Table 5:** The use value index (UVI) and Relative frequency of citation (RFC) of the most commonly used medicinal plants by the local people of different areas of SMR of District Bhimber (AJK), Pakistan (Note: 65 informants participated in this specific analysis).

S No	Names of plants	Common name	Family	Ethnomedicinal Uses	FC	RFC	UV	UVi
					65 informants participated in analysis			
1.	*Acacia arabica* L.	Kikar	Mimosaceae	Healing of wounds, against fever, cough, cold, toothache.	33	0.51	28	0.43
2.	*Acacia nilotica* (Linn.) Delile.	Jangle Kikar	Mimosaceae	For infection in foot, tooth-ache, sexual disorders	28	0.43	21	0.32
3.	*Ailanthus altissima* (Mill.) Swingle	Toon	Simaroubaceae	Relief headaches, rheumatism and skin diseases.	27	0.42	22	0.34
4.	*Albizia julibrissin* Durazz.	Jangle shree	Mimosaceae	Treatment of insomnia, digestive diseases, anticancer, diarrhea.	23	0.35	27	0.42
5.	*Albizia lebbeck* L.	Shree	Mimosaceae	Asthma, kidney diseases, arthritis	21	0.32	18	0.28
6.	*Albizia procera* L.	White shree	Mimosaceae	Treatment of kidney disease, anticancer, digestive disorders.	30	0.46	29	0.45
7.	*Azadirachta indica* (A.) Juss.	Neem	Meliaceae	Wound healing	45	0.69	31	0.48
8.	*Bombax ceiba* L	Simbal	Bombacaceae	Cough, fever, menstrual pain, flu, sore throat	29	0.45	30	0.46
9.	*Broussonetia papyrifera* L.	jangle toot	Moraceae	Tonic, for skin disorders, dysentery, diarrhea.	30	0.46	23	0.35
10.	*Butea monosperma*	Chechra	Papilionaceae	To cure of eye related diseases, diabetes, kidney disorders.	25	0.38	41	0.63
11.	*Cedrela toona* Roxb.	Cedar	Meliaceae	Healing of wounds, tonic, dysentery, skin diseases	22	0.34	24	0.37
12.	*Dalbergia sissoo* L.	Tali	Papilionaceae	Cure skin diseases, abscesses, blood purifier, antiseptic, dental care	20	0.31	26	0.40
13.	*Emblica officinalis* L.	Amala	Euphorbiaceae	Treatment of stomach diseases, diabetes, and kidney disorders, asthma, jaundice	28	0.43	54	0.83
14.	*Eucalyptus citriodora*	Safada	Myrtaceae	Cure cold, cough, flu, pneumonia and fever.	28	0.43	42	0.65
15.	*Eugenia jambolana* L.	Jaman	Myrtaceae	To cure dysentery, anticancer, antioxidant, reduce sugar level.	22	0.34	57	0.88
16.	*Ficus bengalensis* L.	Bohrr	Moraceae	Cure skin diseases, diabetes, tonic, used for toothache	25	0.38	55	0.85
17.	*Ficus elastica* Roxb.	Rubber	Moraceae	For chest infection, constipations, oral infection, gastrointestinal	31	0.48	22	0.34
18.	*Ficus palmata* Forssk.	Phagwar	Moraceae	To cure asthma, digestive, skin diseases, diabetes	29	0.45	37	0.57
19.	*Ficus religiosa* L.	Pipal	Moraceae	To treat dysentery, wound healing, fever, diarrhea.	22	0.34	39	0.60
20.	*Melia azedarach* (L.) Pers.	Darik	Meliaceae	Wound healing, anemia, jaundice	28	0.43	61	0.94
21.	*Ziziphus mauritiana* Lam	Jandi	Rhamnaceae	Anticancer, tonic, blood purifier, fever	26	0.40	45	0.69

These quantitative values depicted the trend of ethnobotanically used plants in respected area of SMR of District Bhimber of AJK. The UVi of various plants species was found to lie within 0.25 to 0.91. Highest value was calculated for *Dalbergia sissoo* (0.91), followed by *Bombax cieba* (0.85), *Butea monosperma* (0.83) while lowest was recorded for *Albizzia julibrissin* (0.25). These values illustrate that *Dalbergia sissoo* plant is more popularly used for different purposes in study area, followed by *Bombax cieba* and *Butea monosperma* in respect of ethnobotanical uses (S1 Table). RFC value was calculated on the bases of the response of the interviewers (who actually participated, who were 65) recorded during survey section. Highest relative frequency was measured for Meliaceae family member *Azadirachta indica* and lowest was measured for *Eugenia jambolana* (RFC = 0.38) belonging to Myrtaceae family. RFC values represent the relative popularity of individual species in study area according to their use. RFC and UV of common plants are listed in (Table 4).

### Relative frequency citation (RFC) and use value (UV) of ethnomedicinal uses trees

Ethnobotanical significance of various plants was calculated by using relative frequency of citation (RFC) and use value index (UVi). These quantitative values depicted the trend of ethnobotanically used plants in respected area. Highest value of UV was calculated for *Melia azedarach* with 0.94 value of UVi and and *Eugenia jambolana* (0.88), then for *Ficus bengalensis* (0.85) and *Emblica officinalis* (0.83). RFC value was calculated on the bases of the response of the interviewers recorded during survey section. Highest relative frequency was measured for Meliaceae family member *Emblica officinalis* (RFC = 0.83) and lowest was measured for *Albizia lebbeck* L. (RFC = 0.28) belonging to family Mimosaceae. RFC and UV of common plants are listed in (Table 5). These indices prove that these plants have much higher ethnobotanical uses and common prevalence in TEMs being promulgated in the study area. The similar research findings have been reported in the previous studies where *Emblica officinalis* and *Eugenia jambolana* have been reported as potential medicinal plants for cure of diabetes and other infirmities in the rural areas of AJK [25, 31].

### Rank order priority of ethnobotanical uses of trees

Rank order priority (ROP) quantitative index is applied to substantiate the EB uses of cited plants by local inhabitants of Samahni area. ROP is interrelated with FL and RPL and often referred as correction factor when FL is different from RPL value. The RPL and FL values along with ROP are presented in (Table 6). ROP values recorded ranges between 5–100, whereas two species *Azadirachta indica* (A.) Juss and *Acacia arabica* L. scored (ROP = 100) value followed by *Acacia nilotica* (Linn.) Delile. (ROP = 83.7) commonly used for timber. While lowest value was recorded for *Ziziphus mauritiana* Lam (ROP = 5.8). The higher ROP values than 50 means that these plants were predominantly used by indegenious people in various cores of life. Plents reported with lower ROP values indecitates that either younger generation has lost interest in EB, they are not readilty avaibale/their number has been reduced in area or there are abundant alternative present in Samahani area (S2 Table). Study divulges that there is need further conservation work in area to protect and conserve its versatile flora and bioculture of the indigenous communities (Table 6). Same previous citation of use of ROP for validation of TEMs and other ethnobotanical uses of wild flora of Azad Kashmir areas has been conducted by Amjad *et al*., and Mehwish *et al*., [25, 31].

**Table 6:** List of ethnobotanical data of indigenous plants depicting highest uses values by FL, RPL, ROP from SMR District Bhimber AJK, Pakistan.

Sr. No	*Names of plants*	Ethnobotanical Use	N	NA	FL	RPL	ROP
1.	*Acacia arabica* L.	Wood	76.0	76.0	100%	1.0	100
2.	*Acacia nilotica* (Linn.) Delile.	Wood	63.0	62.0	97%	0.9	87.3
3.	*Ailanthus altissima* (Mill.) Swingle	Wood	49	44.0	89%	0.8	71.2
4.	*Albizia julibrissin* Durazz.	Wood and for goods	76.0	69.0	90%	0.9	81
5.	*Albizia lebbeck* L.	Fodder, wood	59.0	56.0	94%	0.9	84.6
6.	*Albizia procera* L.	Basket making, wood, fodder.	56.0	51.0	91%	0.9	81.9
7.	*Azadirachta indica* (A.) Juss.	Wood, fodder	78.0	78.0	100%	1.0	100
8.	*Bombax ceiba* L	Cotton and wood.	89.0	76.0	85%	0.8	68
9.	*Broussonetia papyrifera* L.	Fruit, wood, fodder	68.0	59.0	86%	0.8	68.8
10.	*Butea monosperma*	Wood	57.0	41.0	71%	0.7	49.7
11.	*Cedrela toona* Roxb.	Wood, fodder	63.0	42.0	66%	0.6	39.6
12.	*Dalbergia sissoo* L.	Timber	59.0	35.0	59%	0.5	29.5
13.	*Emblica officinalis* L.	Making soap and shampoo, wood	43.0	25.0	58%	0.5	29
14.	*Eucalyptus citriodora*	wood	39.0	21.0	53%	0.5	26.5
15.	*Eugenia jambolana* L.	Fruit, wood	63.0	35.0	55%	0.5	27.5
16.	*Ficus bengalensis* L.	Wood	57.0	28.0	49%	0.4	19.6
17.	*Ficus elastica* Roxb.	Wood	40.0	13.0	32%	0.3	9.6
18.	*Ficus palmata* Forssk.	Wood	65.0	25.0	38%	0.3	11.4
19.	*Ficus religiosa* L.	Wood, thatching	46.0	20.0	43%	0.4	17.2
20.	*Melia azedarach* (L.) Pers.	Wood, fodder	49.0	15.0	30%	0.3	9
21.	*Ziziphus mauritiana* Lam	Wood, fruit, fodder	55	16	29%	0.2	5.8

### Rank order priority of ethnomedicinal uses of trees

Fidelity Level shows that *Morus nigra* L. with maximum FL (51.4%) with (ROP = 34.2) followed by *Melia azedarach* (L.) Pers. and *Ziziphus jujuba* L. with FL (42.8%) were used as antidiabetic and skin diseases, respectively (Table 7, S2 Table, Fig 4). Similar, results have been reported in other parts of Pakistan and AJK in several ethnomedicinal research works demonstrating that local people of mountains areas still dependent on plant to fulfill their life necessities [18, 21, 23].

**Fig 4:** ROP value of indigenous plants species from Shiwalik mountaineous range of District Bhimber AJK, Pakistan.

**Table 7:** List of ethnobotanical data of indigenous plants depicting highest uses values by FL, RPL, ROP from SMR District Bhimber AJK, Pakistan.

Botanical name of plants	Major aliment	Np	FL (%)	RPL	ROP = FL×RPL
*Acacia arabica* L.	Diabetes, skin disease	12	34.2	1.0	34.2
*Acacia nilotica* (Linn.) Delile.	Kidney disorders	05	14.3	0.8	11.4
*Albizia lebbeck* L.	Arthritis	08	22.5	0.6	13.5
*Albizia procera* L.	Kidney diseases	09	25.7	1.0	25.7
*Albizia julibrissin* Durazz.	Anticancer	02	5.71	0.9	5.1
*Azadirachta indica* (A.) Juss.	Wound healing	06	17.1	0.3	5.1
*Broussonetia papyrifera* L.	Cough curing	04	11.4	0.6	6.8
*Bombax ceiba* L.	Cure fever	03	8.57	1.0	8.5
*Butea monosperma* O. Ktz.	Diabetes	08	22.5	0.5	11.2
*Dalbergia sisso* L.	Skin diseases	06	17.1	0.6	10.2
*Emblica officinalis* L.	Stomach diseases	07	20.0	0.9	18.0
*Eugenia jambolana* L.	Dysentery	02	5.71	0.2	20.5
*Eucalyptus citriodora* Parker.	Sore throat, flu	08	22.5	0.4	9.00
*Ficus religiosa* L.	Skin diseases	06	17.1	0.7	11.9
*Ficus carica* L.	Wound healing	09	25.7	0.9	23.1
*Ficus elastica* Roxb.	Asthma	03	8.57	0.3	2.5
*Terminalia belerica* (Gaerten) Roxb.	Heart diseases	05	14.3	0.5	7.15
*Melia azedarach* (L.) Pers.	Malarial fever	15	42.8	0.6	25.6
*Morus nigra* L.	Cough curing	18	51.4	0.9	46.2
*Populus nigra* L.	Cough, fever	03	8.57	1.0	8.57
*Senegalia modesta* Wall.	Muscular pain	08	22.5	1.0	22.5
*Santalum album* L.	Stomach diseases	04	11.4	0.4	4.56
*Ziziphus nomularia* L.	Constipation	08	22.5	0.6	13.5
*Ziziphus jujuba* L.	Blood purifier	15	42.8	0.3	12.8

### Relative importance (RIP) of plants

Numbers of EB plants are also used for medicinal purposes to cure one or more diseases. RLP was calculated to evaluate the potential trading variabilities of cited plants. Potential pharmacological prospective and diseases cured by medicinal plants (MPs) is calculated by relative importance of plants (RIP). Moreover, the multiple uses of these MPs as agricultural products (agro-uses) were also determined to prove their multiple use and popularity in customs of local communities, furthermore export or trade status was also calculated (Table 8, Fig 5). The studies revealed that ethnopharmacological potential was described by using RIP which ranged 11.8 to 50.8. The highest RIP (50.8) was found for *Azadirachta indica* A. Juss. with good number of agro-uses and its seeds and bark were sold or marketed for local markets to prepare herbal therapeutics by indigenous practioners (S2 Table). Followed by *Morus alba* L. with RIP (46.8) and *Albizia julibrissin* Durazz. having (RIP: 46.7) while least RIP value (11.8) was found for *Bombax ceiba* L. It was determined that MPs having less RIP values means that these plants had less medicinal or ethnopharmacological uses in TEMs in the study area. Similar findings have been reported by previous researchers where many trees/plants have been used as source of TEMs [15, 18].

**Fig 5:** Relative importance of tree plants of Shiwalik Mountain Range of District Bhimber AJK, Pakistan.

**Table 8:** Priority ranking (PR) index in the study area from Shiwalik Mountain Range of District of AJK, Pakistan (with destructive threat order: R6 < R5 < R4 < R3 < R2 < R1; 6 is the most destructive value).

Threat Factor	Respondents (R1- R6)						Total	Percentage	Rankings
	R1	R2	R3	R4	R5	R6			
Fuel Source	6	4	4	5	6	6	31	34.4	1^st^
Construction of houses	5	6	5	3	4	5	28	32.2	3^rd^
Decoration and goods	2	3	4	1	2	3	15	16.6	6^th^
Agricultural purposes	2	1	1	3	4	3	14	15.5	7^th^
Timber cutting	4	5	6	4	6	5	30	33.3	2^nd^
Fodder	4	4	3	5	3	6	25	27.7	5^th^
Hedging and Thatching	2	1	3	1	2	2	11	12.2	8^th^
Food	4	3	5	4	5	6	27	30	4^th^

### Priority ranking (PR)

According to the information gathered, it is predicted that extensive use of tree plants for various house cores is very common in the study area. Extensive use of plant and its products causes reduction in respected abundance of plant species, because premature collection flowers, seeds and leaves may lead towards threatening of species. The priority ranking (PR) analysis index determines the abundance status of each ethnobotanically reported tree plants species which predicts the conservation status of the trees. Through VAA and RAA data collected from study area PR value was calculated in order to explore the biotic stresses on plants in study areas. Data was organized into tubular form and destructive order was determined and arranged in six respective orders: 6 < 5 < 4 < 3 < 2 < 1; number 6 represents the most destructive value, as shown in (Table 8). The PR index proved that due to multiple use of one species there is huge stress on its population and it thrills that plant taxon into threatened or endangered zone leading to extinction. It was found that fuelwood use was highest for the tree flora in the study area and it was due to hilly or mountaineous area where on tree wood is used for fuel to cook or heat the room in chilling winters (S1 Table). Pinus was predominantly cut for fuelwood and for timber purposes which generated biotic stress on the plant and it needed urgent work for re-forestation and public-private partnership for conservation of this plant. Similar studies have been reported in the past where indigenous people use or totally rely on wild plants for fuel wood or other daily needs in different areas [1, 25, 32].

This study revealed that trees of the area prevalently used for different necessities of daily life by the indigenous communities. There is common trend for use of botanic or herbal drugs as people have traditional mind and culture having trust on old traditional ethnomedicinal knowledge of the area being received from their forefathers (S2 Table).

### Novelty in ethnomedicinal explorations through Jaccard Index

To explore novel EB and TEMs uses of tree flora of SMR of District Bhimber of AJK, Pakistan, an index named as JI was used. In previous studies conducted on ethnomedicinal and ethnobotanical uses of wild flora it was confirmed that plants /trees were most commonly used in their domestic life. In this study, ethnobotanical results were compared with past works of 25 researchers from Pakistan and other parts of world (S1 and S3 Tables). The values of JI ranged from 1.27 to 13.27; whereas it was found that top three to four similarity or highest JI was recorded for indigenous studies of Azad Jammu and Kashmir or Pakistan as compared with world wide data (S3 Table). This was findings were congruent with previous work of Ishtiaq *et al*., Khan *et al*., and Ajaib *et al*., [18, 25, 32]. This study proves that our research work is novel and valid because it has some similarity for some trees plants while most of them have different TEMs and EB uses (S3 Table), as reported by indigenous communities of SMR of District, AJK.

### Determination of conservation status of tree flora

The research work reveals that as the most areas of SMR are hilly torrents and high lofty mountains where rural dwellers reside in the forest or wild areas. This states that indigenous people of that area primarily cope their daily necessities from environment, using mostly plants and other wild life. Inhabitants of the area relay on natural sources firstly due to lack of advanced form of resources, toxic or side effects and secondly due to high cost of market products (S1 Table). Alongside native inhabitant also believes that herbal medicines are safer for use as compared to pharmaceutical or western medicines. Extensive use of natural sources (wild trees) is causing serious risk to their abundance and growth percentage. It was calculated that wild trees of SMR area are facing high risk factors being triggered due to their extensive and multifarious use by the local people. The extensive conservation work through research and applied form is its key and sustainable solution which can assist ecofriendly approach [13, 26]. The different statistical tools like data matrix ranking and priority ranking prove that wild tree flora is under severe biotic and abiotic stresses, in which former is initiated by man and later one is boosted by climate changes and these findings are congruent with previous work [1, 25, 44]. The lack information and ruthless cutting of trees for domestic or commercial use by the native residents is cause of threat for their occurrence and abundance in the nature. The catastrophes in the nature like earthquake, heavy raining, snow melting or heavy fire with high intensity are other allied factors which are causing threats for the tree biodiversity in the SMR areas of District Bhimber of AJK, Pakistan.

Highest rank of PR is recorded for consumption of trees for fuelwood, followed by wood cutting of plants as source of timber, while lowest is recorded for hedging and thatching (S2 Table). This shows that villagers of study area highly depend upon wood for furniture making, fuelwood, construction, hedging, fencing, fodder, shadow, grazing by lopping the trees and agricultural tools formation. Whereas fresh parts of trees are used for fodder, forage and paving of huts for shadow for summer. This represents key factor that will cause natural flora degradation in study area. These research proves that *Pinus roxburghii* is under severe threat because local people cut it for fuelwood or timber requirement but its revival or growth is very slow and growth from seeds is low ratio. Hence, forest is becoming scarce of pine trees, and deliberate cutting by timber mafia is also accelerating this phenomenon. The other trees like *Melia azedarach*, *Melia azadirachta*, *Butea monosperma*, *Pinus roxburghii*, *Terminalia belerica*, *T*. *chebula*, *Bauhinia variegata*, *Morus laevigata*, *Flacourtia indica* and *Cassia fistula* are under pressure due to cutting for forage or fodder for cows, camels and goats (S1 Table). Their extensive use in making agricultural tools is also exerting pressure on their population which creates pressure. The extensive cutting for different ethnoveterinary uses also one of leading step towards rarity and shortage of population which demands urgent practical actions for conservation studies and to take remedial measures to protect and conserve wild tree flora using *in-situ* and *ex-situ* approaches.

## Conclusions

It is concluded that tree flora of SMR areas of District Bhimber has great impact on daily life of indigenous inhabitants. They obtained many of the basic necessities from these tree species to sustain the life. Many of these taxa are prevalent used in multifarious TEMs and EB uses in different villages and ethnic communities. Relative frequency of citation (RFC) and use value (UV) results illustrated that *Azadirachta indica* plant is more popularly used in study area, followed by *Broussonetia papyrifera* L. while *Eugenia jambolana* L. is least used for ethnobotanical uses.

It was found that Moraceae and Mimosaceae has less biotic pressure rather *Butea monosperma*, *Terminalia belerica* and *T*. *chebula* is being depleted at fast form leading to scarcity of their population. Rank order priority (ROP) quantitative index ranged between 5–100, whereas two species *Azadirachta indica* (A.) Juss and *Acacia arabica* L. scored 100 ROP value followed by *Acacia nilotica* (Linn.) Delile. (with 83.7 ROP value) commonly used for timber. There is huge potential of drug development from many of these tree species. The urgent measures to cultivate in nurseries and then planting them *in-situ* form will assist in reclamation of tree flora which ultimately be beneficial for continuation of provisionary as well as regular services for ecosystems and mankind too.

### Future recommendations

There is dare need to conserve tree flora of the study area because it provides lot of ethnobotanical and folklore herbal therapeutics to indigenous populations for curing different ailments. The study highly recommends strict rules should formulated and applied by government. There is key need to expand the Prime ministers ‘billion’s tree tsunami’ project by involvement of youth in its propagation, cultivation and protection. This will lead towards ‘green revolution’ and make the environment eco-friendly as well as timely raining for good agriculture products and crops.

## Supporting information

S1 Table Ethnomedicinal and Ethnobotanical Uses of Trees of Shiwalik Mountain Range of District Bhimber Azad Jammu and Kashmir, Pakistan. (DOCX)

S2 Table Relative importance of plants and relative pharmaceutical significance of EM/EB Plants from SMR District Bhimber AJK, Pakistan. (DOCX)

S3 Table Comparison among present and previous ethnobotanical studies conducted at local, national, regional and global level by using Jaccard Index (JI). (DOCX)

S4 Table Questionnaire proforma used for collection Ethnomedicinal and Ethnobotanical data. (DOCX)
